The article "Automated Detection of Infection in Diabetic Foot Ulcer Images Using Convolutional Neural Network" was published in 2022. Journal: J Healthc Eng.

# Automated Detection of Infection in Diabetic Foot Ulcer Images Using Convolutional Neural Network

**DOI:** 10.1155/2022/2349849

**Published:** 2022-04-06

**Authors:** J. Yogapriya, Venkatesan Chandran, M. G. Sumithra, B. Elakkiya, A. Shamila Ebenezer, C. Suresh Gnana Dhas

**Affiliations:** ^1^Department of Computer Science and Engineering, Kongunadu College of Engineering and Technology, Trichy 621215, Tamil Nadu, India; ^2^Department of Electronics and Communication Engineering, Dr. N.G.P. Institute of Technology, Coimbatore 641048, Tamilnadu, India; ^3^Department of Biomedical Engineering, Dr. N.G.P. Institute of Technology, Coimbatore 641048, Tamilnadu, India; ^4^Department of Electronics and Communication Engineering, Vel Tech High Tech Dr. Rangarajan Dr.Sakunthala Engineering College, Avadi, Chennai 600062, Tamilnadu, India; ^5^Karunya Institute of Technology and Sciences, Karunya Nagar, Coimbatore 641114, Tamilnadu, India; ^6^Department of Computer Science, Ambo University, Post Box No.: 19, Ambo, Ethiopia

## Abstract

A bacterial or bone infection in the feet causes diabetic foot infection (DFI), which results in reddish skin in the wound and surrounding area. DFI is the most prevalent and dangerous type of diabetic mellitus. It will mainly occur in people with heart disease, renal illness, or eye disease. The clinical signs and symptoms of local inflammation are used to diagnose diabetic foot infection. In assessing diabetic foot ulcers, the infection has significant clinical implications in predicting the likelihood of amputation. In this work, a diabetic foot infection network (DFINET) is proposed to assess infection and no infection from diabetic foot ulcer images. A DFINET consists of 22 layers with a unique parallel convolution layer with ReLU, a normalization layer, and a fully connected layer with a dropout connection. Experiments have shown that the DFINET, when combined with this technique and improved image augmentation, should yield promising results in infection recognition, with an accuracy of 91.98%, and a Matthews correlation coefficient of 0.84 on binary classification. Such enhancements to existing methods shows that the suggested approach can assist medical experts in automated detection of DFI.

## 1. Introduction

Diabetic foot infection is a common complication of diabetes mellitus that requires treatment and is arguably the most prevalent cause of nontraumatic lower extremity amputation. Extended exposure to cold and rainy conditions, soaked feet, alcohol consumption, and smoking are all huge risk factors for developing foot infection. DFI is more common in persons who have heart, renal, or eye problems. DFI is a severe type of injury experienced by people with diabetes [1]. This condition occurs when the bacteria enter the body through the wound. Diabetic foot ulcer (DFU) is not an infection, but it often leads to infection [2]. DFI is caused by bacteria or bone infection in the foot ulcer area, making the wound and the surrounding skin reddish. Diabetic foot infection is cured with the help of antibiotic treatment [3]. If a medical professional does not treat the injury, the infection can spread, leading to pain, discomfort, necrosis, and, in the worst case, amputation. The two major causes of diabetic foot infection are neuropathy and peripheral artery disease (PAD) [4]. Neuropathy (nerve damage) can significantly impair the feeling in the leg [5]. A person unable to feel the pain can risk developing a foot infection. It may allow vulnerable bacteria to enter the body. PAD is another cause of diabetic foot infection; it prevents or slows down the healing process by impairing blood flow. It makes people not feel the initial injury and risk developing foot infection [6]. Physical examination, blood tests, and a Doppler study of the leg diagnose DFI. The physician will look into the foot for signs of foot infection. Therefore, the traditional methods are very costly and time-consuming [7].

The article "Automated Detection of Infection in Diabetic Foot Ulcer Images Using Convolutional Neural Network" was published in 2022. Journal: J Healthc Eng.

Infection should be tested in patients with active DFU and ischemia. Approximately 56% of DFU becomes infected, with 20% of infections resulting in a limb or foot amputation [8, 9]. According to the International Diabetes Federation, 80% of individuals with diabetes mellitus (DM) live in countries with low-income, including India, the world's second-largest diabetes country after China. There are around 69.1 million patients with DM in India with a prevalence rate of 9.3% [10]. To avoid the severe effects outlined previously, a diabetic patient with a “high-risk” foot needs regular doctor visits, expensive medication, and personal sanitary care. As a result, it places a significant financial burden on patients and their families, particularly in underdeveloped nations, where the cost of treatment is high. There are not many computer-aided methods available for the screening of DFI. Recognizing infection in DFU using cost-effective machine learning algorithms is a critical step toward developing a comprehensive computerized DFU evaluation system for remote monitoring. Therefore, it is essential to develop DL algorithms to evaluate foot ulcer images and assess whether patients have infection or no infection.

The recent trends in computer vision (CV) and deep learning (DL) in recognizing foot infection will provide helpful information for the physician for further treatment plans [11]. This research proposes a novel framework for DFI classification based on the motivation from preceding research works. The proposed CNN model integrates features from parallel convolution layers because features contain unique and crucial information about foot infection and for compact representation. The advantage of combining all aspects is that more information about the infection may be gathered and pathologies with comparable appearances to non-infected skin can be treated more effectively. Several CNN models were trained to distinguish between infection and noninfection classes. We then showed that using the proposed model parameters improves overall classification. The works relevant to diabetic foot infection are discussed in Section 2, followed by a discussion of the dataset and the proposed DFINET in Section 3. The collected results are presented in Section 4, followed by a conclusion and future directions in Section 5.

The article "Automated Detection of Infection in Diabetic Foot Ulcer Images Using Convolutional Neural Network" was published in 2022. Journal: J Healthc Eng.

## 2. Related Work

The evolution of DL and CV in medicine has solved most medical imaging and other medical-related problems such as Alzheimer detection, cervical cancer, malarial detection [12], and brain tumour [13]. Infection is defined as at least two classic signs of purulence in DFU. It is difficult to tell from DFU images if diabetic foot infections are present; however, increasing redness in and around the ulcer and colored purulence could be signs of DFI. Blood testing is the gold standard diagnostic test in the medical system. In addition, the images in this dataset were taken after the debridement of necrotic and devitalized tissues, which removes a key indicator of infection in DFU. Rostami et al. [14] proposed the ensemble DL model to determine the wound images from different sources. The proposed model classifies the six classes: normal, normal skin, venous wound, diabetic wound, pressure, and surgical wound. The model achieved 94.28% accuracy in binary classification and 87.70% in multilevel classifications. Kim et al. [15] proposed a model for the prognosis of DFU using thermal images. The ResNet50 model is used as the feature extractor, in which machine learning (ML) algorithms random forest and support vector machine (SVM) are used as a classifier. The model achieved an accuracy of up to 81.1%. Das et al. [16] proposed the CNN architecture with a deep residual block to extract the high-level features, and then the parts are fused with different machine learning algorithms. The logistic regression algorithm achieves an area under the curve value of 96.50%. Hüsers et al. [17] presented the transfer learning method to detect the wound maceration and was able to achieve a recall of 0.69. Carlos Padierna et al. [18] extracted features from infrared images of the upper side of the foot and toes to propose a classification approach for finding PAD and achieved 92.64% using SVM. Adam et al. [19] developed density dual-tree complex wavelet transform in an automated detection method to locate diabetic feet with and without neuropathy. Entropy and texture features were extracted from infrared images and 93.16% accuracy was achieved using a k-nearest neighbour. Alzubaidi et al. [20] developed a CNN model named DFU Queensland University of Technology Net to classify normal and abnormal classes from DFU images. The CNN model is designed by increasing the width and global average pooling, with an F1-score of 94.5% in classifying the class as normal and abnormal. Das et al. [21] proposed the stacked parallel convolution layers to improve the classification performance in classifying normal and abnormal categories. The model achieves an area under the curve value of 0.974. Goyal et al. [22] proposed DL to recognize ischemia and infection from DFU images using the ensemble CNN model and machine learning algorithms. The ensembled model achieved 90% and 73% accuracy in classifying ischemia and infection, respectively. Das et al. [23] proposed a CNN model with different residual blocks consisting of convolution, normalization, leaky rectified linear unit (LReLU), and global average pooling layers. The model achieved better accuracy in classifying ischemia—with an accuracy of 97.8%—than the classification of infection—with an accuracy of 80%—from the diabetic foot ulcer images. Recognition of infection in DFU with light-weight deep learning methods is a significant step toward developing a complete computerized DFU assessment system for remote monitoring in the future due to the high risks of infection in DFU leading to amputation and patient's hospital admission [24]. From the literature, it is found that only two models are available for diabetic foot infection recognition.

The article "Automated Detection of Infection in Diabetic Foot Ulcer Images Using Convolutional Neural Network" was published in 2022. Journal: J Healthc Eng.

DL algorithms for DFI recognition are investigated in the present study, which considers a literature review. To overcome the challenges faced in classifying infection and noninfection due to poor lighting conditions, poor contrast, marks, and skin tone, a new convolutional neural network (CNN) was developed using diabetic foot images from scratch. The following is a list of significant contributions to this work:

1. A 22-layer CNN architecture with convolution layers, batch normalization, ReLU, and a dropout layer is proposed to improve the classification accuracy in predicting infection and noninfection
2. The hyperparameters are studied and fine-tuned for the proposed model to enhance the model's performance

## 3. Materials and Methods

The proposed model is designed to extract the discriminative features efficiently by improving the overall performance in classifying infection and non-infection from diabetic foot ulcer images.

### 3.1. Dataset for the Study

The DFU images with infection are not publicly available, but with the appropriate procedure, they can be accessed [22]. The dataset is assessed once the lead investigator signs a dataset release agreement. The dataset consists of two classes, and each class contains two subclasses, i.e. ischemia versus nonischemia and infection versus noninfection. This study considers infection versus noninfection to improve the overall classification performance. The dataset consists of 5890 images, with 2945 images for infection and 2945 images for non-infection with ground truth labels. A senior physician made the final decision on the ground truth labels. Figures 1(a) presents infection and Figure 1(b) presents noninfection class example images from the dataset.

The dataset found that the images have interclass similarity, poor contrast, and poor lighting conditions. Image augmentation techniques such as sharpening, gamma correction, saturation, and equalization are applied to the dataset to overcome this issue. In the CNN model, the data augmentation technique is also employed to address the problem of overfitting.  Figure 2 shows the augmentation technique applied to the infection classes. In this research, the images in the dataset are resized to 256 × 256 for infection recognition. Each image in the dataset increased by a factor of 5, including the original image. The number of images in the dataset has been increased by 14725 for each class, resulting in 29450 images. In Table 1, the dataset distribution with and without augmentation is given.

### 3.2. Methodology

The overall flow of the proposed methodology is shown in Figure 3. The augmented dataset is split into training (training and validation) and testing sets. The trained model is then tested with a test set, and infection and noninfection are determined using DFU images. The proposed DFINET model is shown in Figure 4 with layer by layer description. 10 convolutional layers, 5 max-pooling layers, 5 normalization layers, and 2 fully connected layers make up the model's 22 layers. The proposed architecture uses the ReLU activation function in the convolutional layer to map negative values to 0 and positive values to a maximum value of *z*. The ReLU function can be determined using equation (1), where *z* is the input of the neuron. The nonlinearity in the dataset is introduced using the ReLU function. Because the negative values are set to 0 in the ReLU function, it is computationally efficient.

(1) $$\begin{array}{c} F\left(z\right)=\text{maximum}\left(0,z\right). \end{array}$$

The normalization layer speeds up the training process by normalizing the feature values using mean and variance across each channel's input. The extracted features from convolutional filters 4, 5, 6, and 7 are concatenated to improve the performance. Concatenated layers take the two blobs and output as a single blob. After feature concatenation, maximum pooling is used to reduce the feature representation and computational complexity. The fully connected layer is integrated with the flattened layer for converting 2-dimensional data to 1-dimensional data. The fully connected layer multiplied the input with the weight value at each node from the flattened layer and provided the output value after adding the bias value. The dropout layer is used in the fully connected layer with a dropout probability ratio of 0.3. The dropout function reduces the overfitting in the proposed model, making the model more general. The SoftMax layer is used to classify the input data as infection or noninfection class by providing the probability of each class. The SoftMax function is calculated using

(2) $$\begin{array}{c} \sigma {\left(z\right)}_{i}=\frac{e^{z_{i}}}{\sum_{j=1}^{k}e^{z_{j}}}. \end{array}$$

Here, *i*=1,2,3,…, *k* and *Z*=(*z*_1_, *z*_2_ … *z*_*k*_) ∈ *Rk*.

The article "Automated Detection of Infection in Diabetic Foot Ulcer Images Using Convolutional Neural Network" was published in 2022. Journal: J Healthc Eng.

Infection and noninfection class patterns that distinguish the two classes are learned using the DFINET model using the training dataset which can aid in enhancing the model's performance.  Table 2 provides the detailed parameters of the proposed model.

### 3.3. Feature Visualization Using Filters

The feature map of the infection and noninfection classes using DFU images is visualized using different convolutions at different layers. The feature map at convolutional layer 1, convolutional layer 2, max pooling_1, and batch normalization_1 layer in the DFINET is shown in Figure 5. The feature visualization maps for convolutional layer activation 2, max pooling layer 2 and batch normalization layer 2 are shown in Figure 6. The feature visualization map of fully connected layers 1 and 2 is shown in Figure 7.

### 3.4. Adam Optimizer

The proposed model uses the Adaptive Moment Estimation (Adam) optimizer as an optimization strategy to update the weights during the training process [25]. Adam uses the running average of both the gradients and second moments of the gradients. Adam is quite computationally effective and requires less memory space. For each parameter, *w*_*j*_ weight update is given by

(3) $$\begin{array}{c} \Delta w_{t}=-\eta \frac{v_{t}}{\sqrt{s_{t}+\varepsilon }}*g_{t}, \end{array}$$

(4) $$\begin{array}{c} w_{t+1}=w_{t}+\Delta w_{t}, \end{array}$$

where *η*=initial learning rate, *g*_*t*_=gradient at time *t*, *v*_*t*_= exponential average of gradients, and *s*_*t*_=exponential average of square gradients.

The article "Automated Detection of Infection in Diabetic Foot Ulcer Images Using Convolutional Neural Network" was published in 2022. Journal: J Healthc Eng.

## 4. Results and Discussion

### 4.1. Comparison of DFINET with Other Models

DFINET, AlexNet, VGG16, and GoogLeNet are experimented with an NVIDIA Quadro RTX6000 using the Caffe DL framework. The obtained dataset is randomly split into three different training and testing sets, provided in Table 3.

The ratio of training and testing is 90:10. The training set is further divided into 70% folds for training and 20% for validation to reduce overfitting in the model. Therefore 21204 (70%) images for training, 5890 (20%) for validation, and 2356 (10%) for the testing phase are used. The model training parameters are set to an epoch of 30, learning rate of 0.0001, batch size of 16, step down policy of 33%, and gamma value of 0.1. The step-down policy is used to reduce the learning rate at every 33% of the training phase. In the DFINET model, the binary cross-entropy function is used as a loss function. DFINET, AlexNet, VGG16, and GoogLeNet are trained using the same parameter. In terms of accuracy (ACC), specificity (SPE), sensitivity (SEN), precision (PRE), F1-Score, and MCC classification metrics, the models are compared with other models described in the literature. The different evaluation metrics are defined as follows:

(5) $$\begin{array}{c} \text{ACC}=\frac{T^{+}+F^{+}}{T^{+}+T^{-}+F^{+}+F^{-}},\\ \text{SPE}=\frac{T^{-}}{T^{-}+F^{+}},\\ \text{SEN}=\frac{T^{+}}{T^{+}+F^{-}},\\ \text{PRE}=\frac{T^{+}}{T^{+}+F^{+}},\\ F1-\text{Score}=\frac{2*\text{PRE}*\text{SEN}}{\text{PRE}+\text{SEN}},\\ \text{MCC}=\frac{\left(T^{+}*T^{-}\right)-\left(F^{+}*F^{-}\right)}{\sqrt{\left(\left(T^{+}+F^{+}\right)*\left(T^{+}+F^{-}\right)*\left(T^{-}+F^{+}\right)*\left(T^{-}+F^{-}\right)\right)}}, \end{array}$$

where *T*^+^ = true positive, *F*^+^ = false positive, *T*^−^ = true negative, and *F*^−^ = false negative.

The training validation plot for the models DFINET, GoogLeNet, AlexNet, and VGG16 is shown in Figure 8. A validation accuracy of 90.80% for DFINET, 79.31% for AlexNet, 77.04% for GoogLeNet, and 86.67% for VGG16 is obtained upon validation at each epoch. The validation accuracy and validation loss are plotted for each epoch. After the models are validated on the validation dataset, they are tested with the testing dataset. The confusion matrix is calculated using the model testing results and shown in Figure 9.

DFINET classification results for correct classification and misclassified images are shown in Figures 10 and 11, respectively. Due to the poor illumination and not-so-steady image-capturing environment, the shadow effect also plays a vital role in classifying infection and noninfection classes. The confusion matrix provides a clear idea about the effective classification performance of the model. The performance values of DFINET, AlexNet, GoogLeNet, and VGG16 models are calculated from the confusion matrix, and SOTA models from the literature are reported in Table 4.

The article "Automated Detection of Infection in Diabetic Foot Ulcer Images Using Convolutional Neural Network" was published in 2022. Journal: J Healthc Eng.

The proposed DFINET performed admirably in classifying infection and non-infection classes. In addition, the proposed models' outcomes are compared to those of the SOTA for infection and noninfection classes. In every classification metric, the DFINET technique surpassed the SOTA performance. The performance shown in Table 4 proves that the proposed DFINET outperforms all the other models. The DFINET model achieves an accuracy of 91.98% in 30 epochs compared to the second-best model VGG16 with 83.11% accuracy. Notably, the DFINET model achieved an MCC value of 0.84, outperforming all the other models with an increased value of 0.18 from the second-best model—VGG16. The MCC provides balanced ratios of the values taken from the confusion matrix. It is more useful in binary classification. The SEN and SPE are the essential performance evaluation metrics in medical imaging applications. The DFINET model yields an SEN value of 90.57% and SPE value of 93.46%, far better than those yielded by VGG16. The results show that the parallel convolution filter and image augmentation are important factors in improving its performance. According to the literature, identifying the infection from the image patches is fairly challenging. The fundamental explanation is that the properties of the infection and noninfection classes are very similar. The wound and its surrounding area get a little reddish when infected, which is a small feature to remember while identifying them. As a result, when we utilize the CNN architecture with parallel convolution filters with better image augmentation to extract more features from multiple convolution filters and when we concatenate them to cover more spread-out clusters from the same image, it allows us to correctly identify them. As a result, the DFINET is shown to be the most effective way to discriminate between infection and noninfection. We have reported the training time of the model in terms of minutes and seconds. The DFINET model takes 36 mins 16 seconds, while the VGG16 model takes 2 hours 45 minutes during training. The DFINET also proves that the model is computationally efficient with better accuracy [26].

With a disease prevalence rate of 0.05, the suggested DFINET model's positive predicted value (PPV) and negative predicted value (NPV) are determined. The PPV and NPV are used to evaluate the DFINET model's diagnostic performance to comprehend the clinical outcome of disease prediction.  Figure 12 illustrates the PPV and NPV values with different probabilities in predicting infection in the DFU images. Although the proposed model does a better job of classifying infection and noninfection, it is essential to consider the model's limitations and future research directions. The collection of more data samples with proper lighting conditions is required.

The article "Automated Detection of Infection in Diabetic Foot Ulcer Images Using Convolutional Neural Network" was published in 2022. Journal: J Healthc Eng.

Furthermore, a generative adversarial network (GAN) can also be explored to generate synthetic data samples to check the model's performance. The DFINET model's understanding in classifying infection and noninfection is visualized using occlusion sensitivity [27].  Figure 13 shows the model's understanding toward the image features used to predict infection and noninfection by the DFINET model.

## 5. Conclusion

In this work, the CNN based model DFINET, the pretrained model VGG16, GoogLeNet, and AlexNet are proposed and trained to classify infection and noninfection classes from the DFU images. The proposed DFINET has provided promising results compared to the pretrained models and models from the literature. Classification of infection and noninfection from the nonstandard images is quite complicated due to the inter-/intra-class similarities and too subtle in foot images. The other factors affect exposure, scars, and texture on the skin. Because texture features provide crucial information about diseases and, as a result, are important for classification (e.g. infection and noninfection), they were used in this study. The DFINET would extract diverse features from a single image as a result of the parallel convolution filters, allowing the proposed model to outperform all other SOTA approaches. When compared to other approaches in classifying infection and noninfection classes, the DFINET model achieved an impressive accuracy of 91.98% and an MCC value of 0.84. The usage of parallel convolution and better hyperparameter tuning are critical in this scenario. Furthermore, the features were important in predicting DFI since they highlighted the difference in skin appearances. The DFINET can help physicians diagnose infection in DFU with reduced time and workload. It further helps make a proper treatment plan for patients to prevent amputation. The performance of these approaches could be enhanced in the future with a more balanced dataset and improved data. The performance of algorithms on this dataset could be improved by further tweaking the hyper-parameters of deep learning methods. The GAN architecture will generate synthetic images to predict the infection in the DFU images. The dedicated web and mobile application for the DFI screening can help in the technological development in telemedicine.

The article "Automated Detection of Infection in Diabetic Foot Ulcer Images Using Convolutional Neural Network" was published in 2022. Journal: J Healthc Eng.

## Figures and Tables

**Figure 1:** Sample images from dataset. (a) Infection. (b) Noninfection.

**Figure 2:** Data augmentation. (a) Original. (b) Sharpen. (c) Gamma correction. (d) Saturation. (e) Elastic transform.

**Figure 3:** Proposed methodology workflow for classifying infection and noninfection.

**Figure 4:** DFINET architecture for classifying infection/noninfection from DFU images.

**Figure 5:** DFINET feature map: (a) input infection image, (b) Conv_1 layer, (c) Conv_2 layer, (d) Pool_1, and (e) Batch Norm_1.

**Figure 6:** DFINET feature map: (a) Conv_2 activation layer, (b) batch Norm_2, and (e) Max Pool_2.

**Figure 7:** DFINET feature map: (a) fully connected layer_1 and (b) fully connected layer_2.

**Figure 8:** Training and validation plot: (a) DFINET. (b) GoogLeNet. (C) AlexNet. (d) VGG16.

**Figure 9:** Confusion matrix from test set. (a) DFINET. (b) GoogLeNet. (C) AlexNet. (d) VGG16.

**Figure 10:** Correctly classified classes. (a) DFINET: actual class = infection; predicted class = infection. (b) DFINET: actual class = noninfection; predicted class = noninfection.

**Figure 11:** Misclassified classes. (a) DFINET: actual class = infection; predicted class = noninfection. (b) DFINET: actual class = noninfection; predicted class = infection.

**Figure 12:** Positive and negative predicted values with a prevalence rate of 0.05.

**Figure 13:** (a) Infection class. (b) Occlusion map of infected class. (c) Noninfection class. (d) Occlusion map of noninfected class.

**Table 1:** Dataset distribution.

Classes	Augmentation	Total images
Infection	Without	2945
Noninfection		2945
Infection	With	14725
Noninfection		14725

**Table 2:** DFINET layer parameter details.

Layer type	Layer parameters Kernel size (KS), number of filters (NF)
Conv_1	KS = 7 × 7, NF = 64
Max_pool_1	KS = 3 × 3, Stride = 2
Conv_2	KS = 3 × 3, NF = 64
Conv_3	KS = 3 × 3, NF = 128
Max_pool_2	KS = 3 × 3, Stride = 2
Conv_4a	KS = 3 × 3, NF = 128
Conv_4b	KS = 1 × 1, NF = 128
Max_pool_3	KS = 3 × 3, Stride = 2
Conv_5a	KS = 3 × 3, NF = 128
Conv_5b	KS = 1 × 1, NF = 128
Conv_6a	KS = 3 × 3, NF = 256
Conv_6b	KS = 1 × 1, NF = 256
Max_pool_4	KS = 3 × 3, Stride = 2
Conv_7a	KS = 3 × 3, NF = 256
Conv_7b	KS = 1 × 1, NF = 256
Max_pool_5	KS = 7 × 7, Stride = 2
FC_1	100
Dropout	Probability = 0.3
FC_1	2
Total number of parameters	14, 895, 440

**Table 3:** Dataset splitting ratio.

Number of images in dataset	Split 1 Train (70%)–test (30%)	Split 2 Train (80%)–test (20%)	Split 3 Train (90%)–test (10%)
29450	Training: 20615 images Testing: 8835 images	Training: 23260 images Testing: 6190 images	Training: 27094 images Testing: 2356 images

The article "Automated Detection of Infection in Diabetic Foot Ulcer Images Using Convolutional Neural Network" was published in 2022. Journal: J Healthc Eng.

**Table 4:** Performance of DFINET in infection classification from DFU images.

Model/classifier	Train/test split	ACC	SEN	SPE	PRE	F1-score	MCC
GoogLeNet	90/10	75.34	73.27	77.82	79.80	76.39	0.50
VGG16	90/10	83.11	81.45	84.95	85.74	83.54	0.66
AlexNet	90/10	76.74	74.96	78.79	80.31	77.54	0.53
DFINET	**90/10**	**91.98**	**90.57**	**93.49**	**93.72**	**92.12**	**0.84**
DFINET	80/20	89.29	88.46	90.63	93.88	91.09	0.77
DFINET	70/30	87.50	92.78	80.28	86.54	89.55	0.74
Ensemble CNN [22]	90/10	72.70	70.90	74.40	73.50	72.20	0.45
Res7Net [23]	90/10	80.00	80.40	80.20	79.70	79.80	0.60
Inception ResNetV2 [22]	90/10	67.60	68.80	66.40	67.20	68.00	0.35
Bayes Net [22]	90/10	63.90	61.90	66.00	65.30	62.20	0.29

## Data Availability

The data used to support the findings of this study are included within the article.
